# COVID-19 Vaccine Acceptance, Attitude, Hesitancy, and Its Associated Factors among Wolaita Sodo University Students: A Mixed-Method Study

**DOI:** 10.1155/2023/2082695

**Published:** 2023-06-01

**Authors:** Afework Alemu Lombebo, Getahun Dendir Wolde, Bezabish Taffese Shomoro, Amelework Gonfa Efa, Mebratu Tila Bscho, Elias Habtu Suleiman, Ashagrie Sintayhu Temesgen, Mahlet Zerfu Arega, Mohammed Suleiman Obsa

**Affiliations:** ^1^School of Medicine, College of Health Science and Medicine, Wolaita Sodo University, Wolaita Sodo, Ethiopia; ^2^School of Anaesthesia, College of Health Science and Medicine, Wolaita Sodo University, Wolaita Sodo, Ethiopia; ^3^Yekatit 12 College of Health Science and Medicine, Addis Ababa, Ethiopia; ^4^Department of Anaesthesia, College of Health Science, Arsi University, Asella, Ethiopia

## Abstract

**Background:**

Countries in the world have been experiencing the ongoing impact and spread of the coronavirus disease (COVID-19) virus pandemic. The health and financial burden of the pandemic has prompted the need for timely and effective vaccination to be considered as the best strategy for controlling disease transmission. However, vaccine acceptability remains an area of concern in developing countries like Ethiopia.

**Objective:**

To assess attitude, hesitancy in the COVID-19 vaccine acceptance, and associated factors among health science students at Wolaita Sodo University.

**Methods:**

A triangulated mixed-method study was conducted. Quantitative data were entered into SPSS Windows version 25 for analysis, and the qualitative data were transcribed using open code version 4.3. A binary logistic regression model was used to establish the association between dependent and independent variables. Adjusted odds ratio (AOR) with a 95% confidence interval (CI) was used to measure the strengths of the association. Thematic approach was used for qualitative data analysis.

**Results:**

A total of 352 students participated in this study. Having family members who were infected with COVID-19, information about COVID-19 vaccine, the need for a vaccine with the level of concern, intention to take COVID-19 vaccine, and academic year were strongly associated with vaccine acceptability. Graduating class and other senior students were about 4 and 2 times more likely to accept vaccination as compared to freshman-year students (AOR = 4.128; 95% CI: 1.351–12.610;*P* = 0.012) and (AOR = 2.195; 95% CI: 1.182–4.077; *P* value = 0.013), respectively. Even if 67% of students had a good attitude towards the vaccine, 56% of the students hesitated to take the vaccine.

**Conclusion:**

The majority of respondents had a constructive attitude towards the COVID-19 vaccine, and only a few of them were vaccinated against the COVID-19 virus. It is of utmost importance to design an evidence-based strategy to increase the uptake of vaccination for healthcare students and other nonhealth science students in universities.

## 1. Introduction

### 1.1. Background

Coronavirus disease (COVID-19) was declared a pandemic by the World Health Organization (WHO) in February 2020, and since then, many countries have been suffering from its spread and impact. Countries in the world have taken public health measures to prevent the spread of COVID-19, such as social distancing, face masks, and vaccination [1]. The virus had an impact on countries all over the globe. There are a total of 380 million confirmed cases and 5.7 million deaths due to COVID-19 at the beginning of 2022. In Ethiopia, the first confirmed cases of COVID-19 were on March 13, 2020. Since then, more than 465,000 confirmed cases of COVID-19 and 7,300 deaths were reported by January 2022 [2].

Although the world has been implementing various COVID-19 prevention strategies, the burden of the pandemic is not notably reduced [3–5]. Owing to significant determination, research, and manufacturing, COVID-19 vaccines were developed shortly afterward [6]. The health and economic burden of the pandemic has caused the need for a timely and effective vaccination to control the spread of the disease [7].

Even though the WHO backed COVID-19 vaccines global access (COVAX) program aims to supply millions of doses for Africa to vaccinate at least 20% of the population, the COVID-19 pandemic continues rapidly [8]. The effectiveness of any vaccination program depends on the awareness, behaviour, and voluntary will of participants [9]. On March 7, 2021, Ethiopians formally began the COVID vaccine as an effective national event after the WHO launched the COVAX program for Africans. Initially, front-line healthcare workers were vaccinated, and later on, the elderly and patients with comorbidities were vaccinated against COVID-19 [10].

University students are informed adults who have higher chances of disseminating the virus but a lower risk of developing COVID-19 complications [11]. Health science students are vulnerable to infectious diseases due to their exposure to clinical practice [12]. A universal evaluation of healthcare professions along with students from 39 countries showed that the rate of hesitancy towards COVID-19 vaccination was 18.9% [13]. Moreover, knowledge gaps regarding vaccine welfare and efficacy have been reported among health science students [14]. Studies conducted in divergent nations have shown that inaccurate information and lack of confidence in vaccines are associated with poor acceptance of vaccines [15, 16]. Despite the success of developing the vaccine against COVID-19, vaccine hesitancy has now become the world's new challenge.

According to the world health organization, vaccination hesitancy is a behaviour that is driven by a variety of circumstances, such as concerns with vaccines or vaccine providers, complacency about the need for a vaccine, and access. People who are vaccine-hesitant are a diverse group who differ in their level of uncertainty regarding certain vaccinations or vaccination in general. Vaccine hesitancy is the result of a complex decision-making process that is influenced by individual and group and vaccine-specific factors, such as communication and media, religion, socioeconomic factors, politics, geographic barriers, and vaccination experience [17–19].

To guarantee effective global vaccination, it is important to inquire about the reasons behind vaccine hesitancy. A handful of studies were conducted on the issue of COVID-19 vaccine acceptance and hesitancy among healthcare workers in Ethiopia, and no notable research has been conducted among Ethiopian university students. This is one of the pioneering mixed-method studies in Ethiopia focusing on university students' intentions to be vaccinated against COVID-19 and could help the government, policymakers, and educators identify students with uncertainty and plan successful actions to enhance tolerance to vaccination. There is scarce information regarding the attitude of university students towards COVID-19 vaccination in the country, particularly in the study area. The study aimed to assess the attitudes, hesitancy, and associated factors of COVID-19 vaccine acceptance.

## 2. Methods

### 2.1. Study Setting

A triangulated mixed-method study was conducted on COVID-19 vaccine acceptance, attitude, hesitancy, and its associated factors among Wolaita Sodo University students from October 1 to November 30, 2021. Wolaita Sodo University endorses various academic programs in health science and medicine. In general, there are Doctor of Philosophy (PhDs), specialties, masters, and undergraduate programs in health science including medicine. It is located 327 km from Addis Ababa, the capital city of Ethiopia, and 160 km from Hawassa, the capital city of the southern nation nationalities and people's regional state. The data showed that a total of 1705 students were registered and learning in health and medicine college during the study period, of which 611 (35.8%) were females and 1094 (64.1%) were males. All Wolaita Sodo University College of Health Sciences and medicine students were our source population while selected students who regularly attended their studies at Wolaita Sodo University College of health science and medicine during data collection time were our study population.

### 2.2. Sample Size Determination

Because research on the adoption of the COVID-19 vaccine among Ethiopian university students has been scarce, the best estimate (P) of 50% was employed in this study. The single population proportion formula was used to calculate the sample size, which had a *P* value of 0.5, a 95% confidence interval, and a margin of error of 5%. Sampling interval K was calculated as being equal to 4.4. To select the study participants, a systematic random sampling method was adopted. Therefore, using the first four students' names from the list they received from the registrar's office and choosing every fourth student based on the order of their names on the list, the lottery method was used to determine the first participant. With a 10% nonresponse rate, the final sample was 382.

### 2.3. Data Collection Tool and Technique

The data collection procedures involve two phases. The first phase is a quantitative survey, which includes a structured self-administered questionnaire, and the second phase is qualitative. Tape records, pens, and notes were used during the interviews. Ten in-depth interviews were conducted and each lasted between 40 and 60 minutes. The quantitative part consists of three sections: part I includes sociodemographic characteristics and students' academic status; part II is about information and knowledge about the COVID-19 vaccine; and part III contains questions about attitude and hesitancy regarding the acceptance of the COVID-19 vaccine. There were 9 attitude statements towards COVID-19 vaccines on a 5-point Likert scale (5 = completely sure, 4 = very sure, 3 = moderately sure, 2 = slightly sure, and 1 = not at all sure) and 5 questions about hesitancy using a 5-point Likert scale (5 = completely likely, 4 = very likely, 3 = moderately likely, 2 = slightly likely, and 1 = not at all likely) regarding concern about COVID-19 vaccines. There were also open-ended questions for the qualitative part of the study assessing attitude and hesitancy. Each study participant was addressed from the registrar list; first, we identified their academic year and departments' and then the questionnaire was given to those selected students for a quantitative study. For the qualitative part, purposively selected students were interviewed until data saturation was declared by the researcher.

### 2.4. Glossary

 
*Freshman Students.* This includes first year university students.
 
*Good Attitude.* The total attitude score of each participant was calculated by summing up the raw score of nine statements. Participants with a score above the mean were considered to have a good attitude.
 
*High Hesitancy*. Participants who scored below the mean were considered to have high hesitancy.
 
*Poor Attitude*. Participants who scored below the mean were considered having a poor attitude.
 
*Poor Hesitancy*. The total score of hesitancy of each participant was calculated by summing up the raw score of five statements. Participants who scored above the mean were considered to have poor hesitancy.
 
*Senior Students*. This includes students who have completed the first year of study.
 
*Vaccine Acceptance*. It is a decision of an individual to accept or refuse a vaccine when presented with an opportunity to vaccinate.
 
*Vaccine Hesitancy*. This means the doubts or concerns towards vaccinations, without referring to actual vaccine receipt.

### 2.5. Data Quality Assurance

To ensure the quality of the data, supervisors and data collectors were trained on the objective of the study, data collection tools, and procedures. Investigators closely monitored the data collection process. The supervisors checked for data completeness and accuracy. Then, the data were coded, computed, and cleaned. Each member of the team checked the content of in-depth interviews. Probing questions were used to promote the free flow of information. Finally, the summary of each interview was repeated for each study participant, and the text of each interview was double-checked by the investigators.

### 2.6. Data Processing and Analysis

Quantitative data were entered into Epi Data Version 4.6.2 and then transported to SPSS Version 25 for analysis. Descriptive statistics and bivariable analysis were performed. Variables that had associations in the bivariable model at *P* < 0.25 were entered into a multivariable logistic regression model to determine the effects of individual variables on patients' perceptions of preoperative fasting guidelines. An adjusted odd ratio (OR) with 95% CI is used to measure the strength of associations. Statistical significance is declared at *P* < 5%. For qualitative analysis, the Amharic audio-recorded interviews were transcribed verbatim into word files and translated into English. All interviews were audio-recorded after taking informed verbal consent, and then a unique identification number was assigned to every interviewee. Audio data were transcribed verbatim and translated into English. The data were first saved in plain text format and then imported into open code software version 4.03 to facilitate coding and categorizing. The investigators read each transcript repeatedly to ensure a degree of standardization and began the coding process. The coded data were compared and organized into groups. Finally, a thematic approach was used to classify and organize the data into key categories. Direct quotes from study participants were narrated word for word.

## 3. Result

### 3.1. Sociodemographic Characteristics

From a total of 382 students, 352 completed the online questionnaire, making the response rate 92%. The majority were aged between 20 and 30 years with a mean age of 23.72 (SD = 3.07). More than half of the students were male 210 (59.7%) and 148 (42%) of the participants were orthodox religion followers. 249 (70.7%) of the participants were senior year students and 149 (42.3%) had an average GPA of between 3.00 and 3.49. Regarding the educational level, the majority 289 (82.1) are undergraduate students (Table 1).

### 3.2. Participants' Experience of COVID-19

The source of information for the COVID-19 virus and vaccine for the majority of the students was social media 177 (50.3%), and 200 (56.3%) of them have adequate information about the vaccine. Among the 352 students, 232 (65.9%) take COVID-19 preventive measures, but only 50 (14.2%) have been vaccinated against COVID-19. 90 (25.6%) of the students' family members were vaccinated for COVID-19 and 45 (12.8%) of the family members were infected with the COVID-19 virus (Table 2).

### 3.3. Intention towards COVID-19 Vaccines

Out of 352 students, 252 (71.6%) intended to receive the vaccine, of which more than one-third, that is, 145 (41.2%) took the vaccine to protect themselves from getting the virus. The other reasons mentioned by the students for being vaccinated were 43 (12.2%) believing that the vaccines are effective and 35 (9.9%) to protect others from getting the virus. The majority of the students, that is, 314 (89.2%) did not oppose the COVID-19 vaccine.

### 3.4. Reasons for Nonacceptance of COVID-19 Vaccine

The majority of the students 302 (85.8%) were not vaccinated against the COVID-19 vaccine, and when asked about the reasons for nonacceptance, the majority of them raised accessibility issues. For example, a 22-year-old female graduating student mentioned the following:

“*I have been asking to be vaccinated but here in the hospital the vaccine is only given to staff and in the community for the elderly and those with chronic illness I wanted to be vaccinated but the vaccine is not accessible to students in our university.*”

The majority of respondents did not want to take the vaccine if it was available, and they gave various reasons. For example, a 22-year-old male senior student stated the following:

“*I do not* want *to be vaccinated because I doubt the effectiveness of the vaccine. I have seen many people who took the vaccine and get infected with the virus repeatedly. So for me, there is no difference between vaccinated and unvaccinated.*”

Of the 352 students, 214 (60.8%) were less likely to take the COVID-19 vaccine; this finding is supported qualitatively because the majority of the study participants stated that they do not want to take the vaccine for the fear of being controlled by the vaccine manufacturers and suppliers (Table 3). For example, a 29-year-old male senior student stated the following:

“*I do not want to be vaccinated because I don't want to be under the control of anyone. I believe that the vaccine has a microchip along with it to control and manipulate human beings in the entire world and I think the vaccines are* fabricated intentionally *for this purpose. In addition to that, I don't trust the suppliers*.”

### 3.5. Student Attitude towards COVID-19 Vaccine

Participants' attitude and hesitancy towards the COVID-19 vaccine were assessed with statements on a 5-point Likert scale. Our study revealed that 67% had a positive attitude towards the COVID-19 vaccine (Table 4). 56% had high hesitancy towards the COVID-19 vaccine (Tables 4 and 5).

### 3.6. Associated Factors towards the Attitude of COVID-19 Vaccine Acceptance

More than two-thirds of 236 (67%) of the students had a positive attitude towards the COVID-19 vaccine. A large number of respondents (197 (56%)) were found to have high hesitancy about being vaccinated against the COVID-19 vaccine. Having a family member with a history of COVID-19 infection, information about the COVID-19 vaccine, the need for a vaccine with the level of concern, intention to take the COVID-19 vaccine, and academic year were strongly associated with vaccine acceptance. Graduating class and other senior students were about 4 and 2 times more likely to accept vaccination as compared to freshman-year students (AOR = 4.128; 95% CI: 1.351–12.610; *P*=0.012) and (AOR = 2.195; CI: 1.182–4.077; *P* value = 0.013), respectively. In addition, students who had a family member with a history of COVID-19 infection were about 3 times more likely to accept vaccination than their counterparts (AOR = 23.317; CI: 1.133–5.754; *P* value = 0.009) (Table 6).

## 4. Discussion

World Health Organization reported vaccine hesitancy as one of the top 10 threats to manage vaccine-preventable diseases [20]. Vaccine hesitancy stems from deep-rooted ideological beliefs and conspiracies [21]. Vaccines from various companies have currently been accepted but their dispensation is limited [22]. Identifying the populations' intent and challenges to vaccination could minimize barriers and increase vaccination. This study determined the acceptance of the COVID-19 vaccine and associated factors among university students. Therefore, identifying acceptance of the COVID-19 vaccine among university students and the factors that determine vaccine hesitancy and attitude towards the vaccine is important in the expansion of efficient health education strategies.

Pieces of research disclosed vaccine acceptability among higher education students in this region. 85.9% of the students were not vaccinated for COVID-19 during the time of investigation; however, our findings show that the likelihood of taking the vaccine was low at 39.2%. This finding is comparable with the study from 37.3% in Uganda [23], 37.4% in Jordan [24], health science students in Egypt (35%) [25], and college students in Addis Ababa, Ethiopia (39.8%) [26]. But the current study finding was lower than findings in Lebanon 87% [27], in China 88.6% [28] in Saudi Arabia 64.7% (27) [29], Qatar (62.5%) [30], in USA 75% (29) [31] and Italy (86%) [32].

Those variations might be due to the variety of types of vaccines available across the world and insight differences towards the vaccine among study groups. Even so, while reconnoitering the reasons behind low acceptance of the vaccine, we note that a significant portion of students reported that they were disquieted about the vaccine's safety, effectiveness, and possible adverse effects, as a similar study was conducted in Saudi Arabia students [29]. The majority of the students stated that the most common reason for being unvaccinated was the accessibility issue of the vaccine and additionally also a limited alternative was available in Ethiopia including the study area at the time of the investigation. In the open-ended section of the questionnaire, one of our students stated that “*I do not want to be vaccinated because I doubt the effectiveness of the vaccine. I have seen many people who took the vaccine and get infected with the virus repeatedly.*” Therefore, it is extremely important to induce them on the vaccine's safety, efficacy, and side effects.

Eventually, in our binary logistic regression, students from rural regions proved to have a 28.3% lower positive attitude towards the COVID-19 vaccine compared to those from the urban regions. Our finding was consistent with the study performed in Bangladesh [33, 34]. More than 85% of Ethiopian people reside in rural areas which remarkably affects their knowledge about COVID-19-related issues. This is because most areas lack adequate internet connections and have poor technology exposure. Evidence suggested that students who had a history of COVID-19 infection presumably had good knowledge and a positive attitude, but our finding shows that only 6.3% of students have been infected with COVID-19 [35].

The academic level of respondents was significantly associated with the multivariate analysis. Graduate class students had a higher positive attitude towards the COVID-19 vaccine than freshman students. This differs from the findings of Bangladeshi [33], Iran [36], and Bangladeshi [34]. Graduate class students had adequate information because they get information from different sources during the COVID-19 era than freshman students.

Our finding indicates that 50% and 41.5% of the students knew about the COVID-19 vaccine through social media and mass media, respectively, which corroborates a prior study conducted by Mannan DKA [37]. The majority of university students consume the contents of social media which has increased their exposure to COVID-19 facts. Following COVID-19, many people turned to social media for information and guidance. This behaviour has both positive and negative aspects. These range from the spread of misinformation to social media's indispensable role in the dissemination of accurate information and mental health education. The ease of access to information is a significant benefit of social media and other digital platforms. This ease of access provides numerous opportunities for education. However, the spread of misinformation on social media and other digital platforms has been identified as a public health threat on par with the virus itself [38–40]. More than half of the students had adequate knowledge about the vaccine but this finding is worrisome as 43.2% of respondents had inadequate information. Since all students are at a higher institution with sufficient scholastic qualifications, it was expected that they possess decent knowledge about the vaccine. This symbolizes a lack of self-awareness, which results in a paucity of knowledge about the vaccine [41].

In terms of demographic variables, around 43.8% of the college students in our sample stated that they were not encouraged by the healthcare providers to be vaccinated against COVID-19. This result calls for the need for every healthcare provider to work on their patients as people tend to listen more to the counselling given by healthcare workers [28, 42].

In our study, 56.0% of the students reported hesitancy to take the COVID-19 vaccine which is lower than a study done in the general population of Ethiopia (68.6%) (38) and similar studies done in Uganda (62.7%) [23], and the finding of Latkin CA reported 60.6% [43]. This variation between our study participants and the general population might be due to the relatively higher level of knowledge and access to a wide range of information of university students. However, it is higher than a study done on university students in the USA (47.5%) (40), Egypt (19.4%) [25], and Northwest China (22%) [44]; this can be due to the differences in the vaccine types provided for different nations and misinformation about the vaccine.

Similarly, 65.9% of the students who thought of other alternative self-protection behaviours other than vaccination were highly likely to hesitate about vaccination. The experience of COVID-19 vaccine hesitancy and denial among health science students is concerning [45, 46]. Shreds of evidence revealed that this might be because of inaccurate information [46]. Convincing a good number of higher education students is, therefore, of public health importance [13]. Higher education centres have to promote educational and social campaigns to shed light on the importance of the COVID-19 vaccine to change the behaviour of their students [44].

Our study included nearly proportional groups of male (59.7%) and female (40.3%) students. While this study was conducted in October, COVID-19 infection was rapidly increasing in Ethiopia. About 71.6% of the students intended to take the COVID-19 vaccine if the vaccines were available. This is higher than a study done on the population of Ethiopia (31.4%) (38), Saudi Arabia (64.7%) [29], and Jordan (36.8%) [47], and it was consistent with the percentage reported by a global survey that included participants from 19 countries (71.5%) [28] and a study done in Bangladeshi (72%) [34]. Even though supported by the previous study, it is much lower than similar studies done in Ecuador (97%) [48] and China (91.3%) [49].

Nowadays, people's attitude towards the COVID-19 vaccine is changing because most of them want to end the pandemic. As a result, the intention to take the vaccine and vaccination rate is increasing. Though most students had the desire to receive a vaccine, 10.8% of them refused to take it. Willingness to protect them from the disease (41.2%) was the most mentioned motivation to take the vaccine.

### 4.1. Limitation of the Study

In the qualitative part of the study, participant responses might have been influenced by the interviewers' own biases and the presence of the interviewer might have in turn affected the participant response. The qualitative findings of this study belong to those interviewed, hence may not be generalizable and transferable. However, we used methodological and investigator triangulation to increase the credibility and generalizability of the findings. Although efforts were made to ensure fidelity to the context during translation, analysis, and interpretation, errors during translation and interpretation might exist.

## 5. Conclusion

In the present study, having family members with a history of COVID-19 infection, information about the vaccine, the need of vaccine with the level of concern, intention to take COVID-19 vaccine, and academic year were strongly associated with vaccine acceptability. The majority of students had a positive attitude towards the COVID-19 vaccine, but only a few were vaccinated for COVID-19. More than half of the students were hesitant to take the vaccine and were still worried about vaccine safety, effectiveness, and adverse effects. These concerns continue to be major factors affecting students' attitudes towards the COVID-19 vaccine acceptance. It is necessary to plan an evidence-based program to encourage the rate of vaccination of health science students. Creating trust towards the COVID-19 vaccine among university students via the dissemination of accurate messages is the key to the triumph of vaccinating many. Future research is needed to further investigate reasons behind COVID-19 vaccine acceptance and to assess the effectiveness of promotion strategies.

## Figures and Tables

**Table 1:** Sociodemographic characteristics of students in Wolaita Sodo University, College of Health Sciences and Medicine, Southern Ethiopia, 2022 (*N* = 352).

Variables	Categories	Frequency	Percent (%)
Sex	Male	210	59.7
	Female	142	40.3

Place of birth	Urban	233	66.2
	Rural	119	33.8

Religion	Orthodox	148	42
	Protestant	128	36.4
	Muslim	33	9.4
	Catholic	25	7.1
	Others	18	5.1

Marital status	Married	35	9.9
	Single	317	90.1

Mother's educational status	No formal education	110	31.3
	Primary education	113	32.1
	College and above	129	36.6

Father's educational status	No formal education	64	18.2
	Primary education	105	29.8
	College and above	183	52.0

Academic year	Freshman	18	5.1
	Senior	249	70.7
	Graduating	85	24.1

Department	Public health officer	51	14.5
	Anesthesia	62	17.6
	Pharmacy	43	12.2
	Medical laboratory	38	10.8
	Midwifery	32	9.1
	Nursing	63	17.9
	Medicine	62	17.6
	General MPH	1	0.3

Average GPA	<1.99	2	0.6
	2.00–2.49	22	6.3
	2.5–2.99	95	27.0
	3.00–3.49	149	42.3
	3.5–4.00	84	23.9

Living arrangement	Off-campus	305	86.6
	On-campus	47	13.4

Educational level	Undergraduate	289	82.1
	Postgraduate	63	17.9

**Table 2:** Participants' experience of COVID-19, Wolaita Sodo University, 2021 (*n* = 352).

Variables	Categories	Frequency	Percent (%)
Source of information about the COVID-19 virus and vaccine	Social media	177	50.3
	Mass media (TV, radio)	146	41.5
	Health professional	25	7.1
	Friends	4	1.1

Encouragement by a health care provider to take COVID-19 vaccine	Yes	198	56.3
	No	154	43.8

Have adequate information about COVID-19 vaccine	Yes	200	56.8
	No	152	43.2

Suffering from chronic illness	Yes	55	15.6
	No	297	84.4

Usage of COVID-19 preventive measures	Yes	232	65.9
	No	120	34.1

Family member infected with COVID-19	Yes	45	12.8
	No	307	87.2

Have you been infected with COVID-19?	Yes	22	6.3
	No	330	93.8

Have you been vaccinated for COVID-19?	Yes	50	14.2
	No	302	85.8

Family members vaccinated for COVID-19	Yes	90	25.6
	No	262	74.4

Level of concern of infecting others with COVID-19	Strongly concerned	198	56.3
	Neutral	114	32.4
	Not concerned	40	11.4

Need of vaccine with the level of concern	Yes	243	69.0
	No	109	31.0

Do you oppose vaccination?	Yes	38	10.8
	No	314	89.2

Likelihood of being vaccinated against COVID-19	Highly likely	138	39.2
	Less likely	214	60.8

**Table 3:** Reasons for nonacceptance of COVID-19 vaccine, Wolaita Sodo University, 2021 (*n* = 352).

Reasons for intention to take scientifically approved vaccine	Frequency	Percentage (%)
To protect myself from getting COVID-19	145	41.2
To protect others from the virus	35	9.9
I believe that vaccines are effective	43	12.2
Health workers' recommendation	20	5.7
I am at high risk	19	5.4
Job requirement	2	0.6
Others	88	25.0

**Table 4:** Attitude statements towards COVID-19 vaccine, Wolaita Sodo University, 2021 (*n* = 352).

Statements	Number of participants (%)				
	Complete sure	Very sure	Moderate sure	Slightly sure	Not at all sure
I do not get vaccinated for personal freedom of choice	34 (9.7)	24 (6.8)	29 (8.2)	91 (25.9)	174 (49.4)

I do not believe in the safety of vaccines	25 (7.1)	30 (8.5)	68 (19.3)	70 (19.9)	159 (45.2)

Do not vaccinate for religious reason	25 (7.1)	23 (6.5)	47 (13.4)	60 (17.0)	197 (56)

Worried about side effects of the vaccine	43 (12.2)	75 (21.3)	118 (33.5)	68 (19.3)	48 (13.6)

Do not need a vaccine for my risk level	18 (5.1)	42 (11.9)	58 (16.5)	87 (24.7)	147 (41.8)

Worried about allergic reaction to the vaccine	19 (5.4)	34 (9.7)	65 (18.5)	82 (23.3)	152 (43.2)

I do not trust physicians who recommend the vaccine	24 (6.8)	21 (6.0)	54 (15.3)	67 (19)	186 (52.8)

Bother me that no long-term studies have been not done on the vaccine	88 (25)	76 (21.6)	82 (23.3)	60 (17.0)	46 (13.1)

It protects me from getting COVID-19 infection	53 (15.1)	46 (13.1)	95 (27.0)	101 (28.7)	57 (16.2)

Over all attitude	Bad attitude	116	33%		
	Good attitude	236	67%		

**Table 5:** Hesitancy towards COVID-19 vaccine, Wolaita Sodo University Students, 2021 (*n* = 352).

Statements	Number of participants (%)				
	Completely likely	Very likely	Moderately likely	Slightly likely	Not at all likely
How sure are you to take a vaccine, if it is available?	33 (9.4)	66 (18.8)	74 (21.0)	104 (29.5)	75 (21.3)

How sure are you to complete the second dose of vaccine despite getting side effects?	18 (5.1)	33 (9.4)	82 (23.3)	102 (29.0)	117 (33.2)

How sure are you to complete a second dose vaccine, despite the lack of long term studies on vaccine?	20 (5.7)	47 (13.4)	95 (27.0)	104 (29.5)	86 (24.4)

*Studies on vaccine*					
How sure are you that you will have access to the COVID-19 vaccine if it is available?	17 (4.8)	51 (14.5)	90 (25.6)	138 (39.2)	56 (15.9)

How likely are you to take the COVID-19 vaccine, if it is available?	37 (10.5)	46 (13.1)	90 (25.6)	107 (30.4)	72 (20.5)

Hesitancy	High hesitancy		197		56
	Poor hesitancy		155		44

**Table 6:** Factors associated towards COVID-19 vaccine acceptance, Wolaita Sodo University students, 2021 (*n* = 352).

Variable	Category	Frequency	AOR at 95% CI	*P* value
Average GPA	<1.99	2 (0.6%)	—	—
	2.0–2.49	22 (6.3%)	0.387 (0.112–1.343)	0.135
	2.5–2.9	95 (27%)	1.052 (0.553–2.002)	0.878
	3.0–3.49	149 (42.3%)	0.966 (0.543–1.716)	0.905
	3.5–4.0	84 (23.9%)	1	1

Academic year	Graduating	18 (5.1%)	4.128 (1.351–12.610)	0.014
	Senior	249 (70.7%)	2.195 (1.182–4.077)	0.012
	Freshman	85 (24.1%)	1	1

Marital status	Single	317 (90.1%)	1.236 (0.493–3.101)	0.651
	Married	35 (9.9%)	1	1

Place of birth	Rural	233 (66.2%)	1.380 (0.835–2.281)	0.209
	Urban	119 (33.8%)	1	1

Have adequate information about COVID-19 vaccine	Yes	200 (56.8)	0.502 (0.274–0.921)	0.026
	No	152 (43.2)	1	1

Need of vaccine with the level of concern	Yes	243 (69)	0.281 (0.14–0.565)	*P* ≤ 0.001
	No	109 (31)	1	1

Family member infected with COVID-19	Yes	45 (12.8)	3.317 (1.133–5.754)	0.009
	No	307 (87.2)	1	1

Intention to take COVID-19 vaccine	Yes	252 (71.6)	0.399 (0.174–0.917)	0.03
	No	100 (28.4)	1	1

## Data Availability

The data used to support the findings of this study are available from the corresponding author upon request.

## Abbreviations

AOR: Adjusted odds ratio
WHO: World Health Organization
COR: Crude odds ratio
CI: Confidence interval
GPA: Grade point average
WSU: Wolaita Sodo University.
